# A Comparative Study between Proximal Femoral Locking Plate and Multiple Cannulated Screws for Fixation of Femoral Neck Fractures in Young Adults

**DOI:** 10.1155/2022/1286419

**Published:** 2022-02-16

**Authors:** Jun Zhang, Yunqiang Zhuang, Li Dai, Dichao Huang

**Affiliations:** Department of Orthopaedic Surgery, Ningbo No.6 Hospital, Ningbo 315040, China

## Abstract

**Objective:**

To compare the clinical effect of proximal femoral locking plate (PFLP) versus multiple cancellous screw (MCS) for FNF.

**Methods:**

FNF patients were treated with the PFLP implant or multiple cancellous screws (MCSs). Patient has been followed up for at least 12 months after surgery nonunion, and the occurrence of complications, femoral neck shortening, fracture healing time, and Harris hip score were recorded and compared.

**Results:**

77 FNF patients were treated with the PFLP (36 patients) or MCS (41 patients). The sex, age, side of the injured limb, type of Garden fracture, time from injury to surgery, and fracture healing time of two groups patients were comparable. The operation time and intraoperative blood loss in the PFLP group were worse than those in the MCS group. Two patients with the PFLP (5%) and nine patients (21%) with the MCS experienced cut out of the lag screw or avascular necrosis of the femoral head or nonunion and received hip replacement. However, the number of fluoroscopies in the PFLP group was significantly lower than that in the MCS group. Additionally, the femoral neck shortening and Harris hip score were all strongly better in the PFLP group than in the MCS group.

**Conclusions:**

Compared with the MCS, PFLP treatment for FNF in young adults can decrease the fluoroscopy times, improve hip functional recovery, and reduce the complications rate and femoral neck shortening.

## 1. Introduction

Femoral neck fracture (FNF) is one of the most common types of fractures, and the lower limb of patients cannot move and the quality of life is severely affected [1]. Osteoporosis is the main cause of FNF, and FPF patients are mainly manifested as lower limb shortening and abduction. Elderly patients accounted for the largest proportion, but with the development of the economy and continuous advancement of the industrialization process, the proportion of young and middle-aged FPF patients has been increasing year by year in recent years [2]. The patient's age, physical condition, and fracture status have an impact on the choice of FNF treatment options, so choosing an appropriate treatment option is very important for FNF patients. However, maintaining the femoral head may cause many complications, such as implant penetration and nonunion. What is more worrying is that the current internal fixation schemes for the treatment of FNF cannot avoid the above complications [3].

In the plate fixation, the PFLP has its own advantages, including the ability to anatomically fit the proximal femur, and the locking screw can be fixed to the femoral head and femoral neck at multiple points [4, 5]. Since 2016, a new internal fixation setting was used to treat FNF in young adults during the operation of the PFLP. In the present study, we compared the clinical effects of the PFLP and multiple cancellous screw (MCS) on treating FNF patients. To our best, the present is the first attempt at comparing the complications and function after the use of the PFLP versus the conventional fixation method.

## 2. Methods

77 FNF patients from February 2016 and December 2019 in our hospital were enrolled in our study. Inclusion criteria: age from 18 to 65 years, fresh FNF (less than <2 weeks), close reduction, follow-up for more than 12 months, and no other fractures in the ipsilateral limb. Exclusion criteria: time of fractures >2 weeks, severe multiple traumas, pathological fractures, combined osteoarthritis and postdysplastic deformities, and follow-up < 12 months. 77 FNF patients were randomly divided into the PFLP treatment group (*n* = 36) and MCS treatment group (*n* = 41). All patients were treated by doctors Z J and ZYQ.

In group 1, 9 patients are caused by falls, 16 traffic accident, and 11 sport injuries. In the group 2, 15 patients are caused by falls, 17 traffic accident, and 9 sport injuries. The Garden classification in group 1, Garden II is 8, Garden III is 16, Garden IV is 12. In group 2, Garden II is 15, Garden III is 20, and Garden IV is 6.

Follow-up: 6 weeks, 3, 6, and or longer after discharge; follow-up time is 12–36 months, average was (15.6 ± 10.0) months; follow-up method: patients return to the hospital for evaluation.

### 2.1. Surgical Protocol

After the patient was anesthetized, a tractor was used for closed reduction, and all the following operations are carried out under the fluoroscopy of the C-arm X-ray machine. We used the Garden alignment index to assess the effect of closed reduction. After 3 failed reductions, the patient was performed open reduction.

For PFLP treatment, starting from the greater trochanter of the femur, make a laterally downward longitudinal incision of about 6-7 cm and make a layer-by-layer incision to expose the greater trochanter of the femur and the lower outer cortex. The new internal fixation setting was applied in the PFLP operation, as shown in Figure 1. Place the 5-hole proximal femoral nail locking plate on the greater femur. The inferior and lateral sides of the tuberosity are slightly posterior, and under the guidance of the locking sleeve, three guide pins are placed in sequence at the proximal end of the femoral neck fracture for temporary fixation. Approximately 0.5–0.7 cm below the cartilage is suitable.

According to the measurement, select a hollow locking nail with a suitable length, place it in sequence, and then insert the locking screw with the fourth hole perpendicular to the femoral shaft, and again, C-arm X-ray and optical-mechanical fluoroscopy confirmed that the fracture reduction and internal fixation were in good position, as shown in Figure 2.

For MCS treatment, fixations were done with cannulated screws. Insert the guide wire above the small rotor and make sure it is in the center position by X-ray. Then, guide wires or drills were inserted around it up to the subchondral bone of the femoral head as an inverted triangle.

### 2.2. Postoperative Management and Evaluation

All patients receive the same treatment. In brief, patients were injected for the low-molecular-weight liver and kidney to prevent deep vein thrombosis, exercised on the bed on the 2nd day after surgery, and performed contact weight-bearing exercise on the 6th week after surgery.

The operation time, intraoperation blood loss, fracture healing time, osteonecrosis of femoral head, infection, failure of fixation, nonunion, reoperation, femoral neck shortening, and Harris hip score were recorded and compared. Nonunion was diagnosed as lack of union after 6 months of follow-up. Criteria for avascular osteonecrosis of femoral head: according to FICAT staging, the X-ray shows the femoral head density changes, including sclerosis, cystic change, uneven density, and even the collapse of the femoral head trapped. ZJ, ZYQ, and HDC are responsible for evaluating qualitative assessment of shortening using the X-ray machine. We detected the shortening of femoral neck as previously described and analyzed the repair effect of fractured hip on X-ray film by the overlap method. The degree of shortening of the femoral neck was assessed by Zlowodzki M et al. [6]. Garden's index [7] was used to evaluate the quality of fracture reduction, and Harris hip score was used to assess the functional outcome [4].

### 2.3. Statistical Analysis

SPSS 19.0 (SPSS, Chicago, IL, USA) was used to analyze the data in this study. Mean ± standard deviation was used to show the measurement data, and the measurement data are analyzed using Student's *t*-test. Categorical data were used to analyze by the *χ*^2^ test or Fisher's exact probability method. *P* < 0.05 was indicated significantly different.

## 3. Results

77 FNF patients were included in the present study, and the time of follow-up was 12–36 months. The sex, age, side of the injured limb, type of Garden fracture, time from injury to surgery, and fracture healing time of two groups patients were comparable, as given in Table 1.

As given in Table 2, intraoperative blood loss has a significant difference within the two groups (36 ml PFLP vs. 13 ml MCS). The operative time is a little longer in the PFLP than in the MCS (53.05 min PFLP vs. 47.78 min MCS, *P* < 0.05). Two patients with the PFLP (5%) and 9 patients (21%) with the MCS were diagnosed with postoperative complications. The time to implant failure in the PFLP group and MCS group was 2.3 months and 3.2 months, respectively. The number of PFLP fluoroscopy was lower. In the PFLP group, femur shortening is 27 (75%), 6 (16.67%), and 3 (8.33%) for mild, moderate, and severe, respectively, while 26 (63.42%), 16 (39.02%), and 9 (2.2%) in the MCS group, respectively. The fracture healing time in PFLP and MCP groups was (4.82 ± 2.25) months and (4.52 ± 1.76) months, respectively. There was 1 (2.78%) case each of nonunion and crew-out, and 2 (5.56%) cases underwent total hip arthroplasty. At the same time, there were 3 (7.31%) cases, 2 (4.88%) cases, and 4 (9.76%) cases of nonunion, osteonecrosis, and screw-out in the MCS group, respectively. At the last follow-up by outpatient, the Harris hip score of the PFLP group was better (93.88 ± 7.26) vs. (87.92 ± 10.34).

## 4. Discussion

Recently, the incidence of FPF is increasing year by year with the aging of the population and the increase of traffic accidents. At present, femoral neck fractures account for 3.6% of total fractures and 48–54% of hip fractures [8]. Due to the high incidence of nonunion of fractures and avascular necrosis of the femoral head after FPF in the past, femoral neck fractures were once called “unresolved fractures.” With the advancement of imaging technology and equipment, internal fixation materials and design, treatment concepts, and surgical techniques, the therapeutic effect of FPF has been significantly improved. However, the incidence of nonunion of fractures and avascular necrosis of the femoral head is still high [9]. The patient's age, health status, fracture type, and treatment method affect the prognosis of fracture patients, and closed reduction cannulated screw internal fixation can be used for young and middle-aged patients and elderly patients with poor physiological conditions. Previous studies have shown that the failure rate of the treatment of fractures with head preservation and femoral neck is higher, some of which exceed 40% [10]. Some FNFs cannot be accurately reduced and fixed due to two reasons [11]: on the one hand, the surgeon is not experienced enough to fully grasp the reduction skills, and the intraoperative C-arm X-ray fluoroscopy is not enough to show the direction and degree of fracture displacement in detail. On the one hand, the fracture displacement is serious, and it is difficult to perform anatomical reduction using conventional reduction techniques. In the past, such fractures often required open reduction and fixation. The trauma was large, and the postoperative fracture nonunion and avascular necrosis of the femoral head had a high incidence of complications. Closed and precise reduction of femoral neck fractures is the key to the success of internal fixation surgery, which helps to reduce the incidence of postoperative complications such as nonunion of fractures and avascular necrosis of the femoral head, and a good treatment plan can reduce the incidence of femoral head necrosis. Therefore, an appropriate treatment plan is very important for young and middle-aged FNF treatment.

At present, there are many types of FPF internal fixation for surgical treatment, which are generally divided into intramedullary fixation devices and extramedullary nail-plate fixation devices. Intramedullary fixation systems include the gamma nail (GN), percutaneous compression plating (PCCP), and PLFP. How to choose the right internal fixation has always been a controversial topic, especially for young and middle-aged patients, which kind of internal fixation has more advantages [12]. Three cancellous screws have been proven to be effective in treating FNF, helping to tighten the fractured ends and promote fracture healing, and this program is simple to operate and has low trauma to patients. In addition, the three cancellous screws can also help reduce the pressure in the joint cavity. However, more and more shortcomings are exposed, that is, the three cancellous screw treatment program has higher complications. The main reason is that the design length of the cancellous screw cannot maintain the length of the femoral neck due to bone resorption during the fracture healing process, specifically the tail of the screw is located outside the trochanter of femur, and the risk of internal fixation loosening is higher [13].

Unstable fractures of the proximal femur have always been a difficult problem in clinical treatment due to difficulty of reduction and fixation. The clinical prognosis of patients also depends on the restoration of the femoral force line during the operation and healing of the fracture [14]. Compared with intramedullary fixation, plate fixation has certain theoretical advantages, including obtaining and maintaining anatomical reduction of fractures and avoiding iatrogenic damage to the abductor muscles. In plate fixation, the PFLP has its own advantages, including the ability to anatomically fit the proximal femur, and the locking screw can be fixed to the femoral head and femoral neck at multiple points [15]. More important was that the PFLP reduced the risk of complications and resisted femoral neck shortening. Therefore, stable mechanical support was one of the advantages of the PFLP.

At present, there are many treatment options for cervical and femoral fractures, but the results are not stable. In the present study, the fixation failure rate of the PFLP group (2.94%) was lower than that in the MCS group (8.82%), and the shortening of femoral neck and Harris hip score at the last follow-up in the PFLP group were significantly better than that in the MCS group (*P* < 0.05).

The PFLP is a kind of the nail plate system, and the biggest difference from the anatomical plate is that the plate can be tightly combined with the locking screw through the threaded locking hole. After the screw is screwed into the bone, the fracture block, locking screw, and the locking plate form a mechanically conductive whole, which meets the requirements of both the correction of the rotation force and the weight bearing of the proximal femur. This PFLP system has many advantages. For example, the three locking screw nuts were designed for locking, but the locking screw nuts also can compress through placing lag cancellous screws. Two 7.3 mm cancellous lag screws can act as a pressure on the fracture line and one 7.3 mm locking cancellous screw can combine the plate with the femoral head forming an angular stabilization. Previous studies have found that the PFLP can reduce the incidence of complications such as failure of fixation and shortening of the femoral neck [13] and can also could help to disperse stress through the plate to help reduce the single nail looseness caused by excessive stress. According to the anatomical characteristics of the femoral neck, the angle between the direction of the three hollow screws and the femoral shaft is designed to be 130°, and the three holes are designed to have 20° tuning, ensuring the accuracy of cancellous screws placement. As a fixed angle device, the PFLP helps to adjust the screw placement direction and spacing.

Previous studies have found that fixation with a nail-plate system was very suitable for treating the patient with Garden type III/IV and Pauwels type II/III FNF; due to these, patients have poor biomechanical stability and high failure rate of internal fixation [16]. Therefore, we assume that insufficient mechanical stability causes the MCS treatment effect to be unsatisfactory.

Biomechanical experiments have showed that the PFLP system not only has the advantages of simple operation, clear fracture exposure, good fracture reduction, and better antirotation but also strong stability. To our best, the study of the PFLP to treat intracapsular hip fractures was few, and only studies by Parker et al. [14] and Lin et al. [17] were similar to that in our study. However, there was no control group in the previous study. In our study, the nonunion rate in the PFLP group was lower than previous studies. Moreover, our results overturn some previous conclusions [18]; the PFLP is not suitable for intracapsular femoral fractures due to the high failure rate of PFLP treatment. The reasons for the differences are as follows: differences in patients, implants, follow-up time, and surgical quality. In our study, the proximal three screws consisted of two lag cancellous screws and one locking cancellous screw; the two lag cancellous screws act as a pressure on the fracture line and the locking cancellous screw strengthen the angle stability of plates and screws. The fracture healing time of two groups were comparable, and the Harris hip score was higher.

FNF is likely to be shortened because the fractured end is generally thicker at one end and thinner at the other end. When a fracture occurs, it is likely that a thinner distal end is inserted into a thicker proximal end due to traumatic impact. This type of fracture is clinically called insertion sexual fractures, so that a certain shortening may occur after the fracture has healed [15]. In this study, we found that compared with the MCS group, there was lower incidence of femoral neck shortening. However, compared with the PFLP group, femoral neck shortening in the MCS group was worse, due to insufficient antishortening performance. The incidence of femoral neck shortening was high after hollow screw fixation [19]. The reason for our analysis may be that the PFLP system fixes the femoral head and neck, with strong holding force and obvious stress dispersion, preventing the screw stress concentration from cutting the femoral head and neck [20], and the tension hole can achieve the effect of compressing the fracture end and the fracture block to ensure the reduction requirement [21].

## 5. Conclusion

Herein, results showed that PFLP treatment for FNF in young adults can decrease the fluoroscopy times, improve hip functional recovery, reduce the complications, and minimize femoral neck shortening. The limitations of this study must be demonstrated: selection bias and small sample size and short follow-up time. In the future, the multicentral, random-controlled, and long-term follow-up trials should be conducted to confirm the validation of the results.

## Figures and Tables

**Figure 1:** The newly designed cannulated screw locking plate used in this study.

**Figure 2:** A 46-year-old male patient with a left Garden type-3 femoral neck fracture treated by the PFLP. (a) Preoperative X-rays and CT. (b) Satisfactory reduction on the first day postoperatively. (c) Fracture partial healing by the second month postoperatively. (d) Fracture healing and stable internal fixation by the fourth month postoperatively.

**Table 1:** Patient demographics between the PFLP and MCP groups.

	PFLP	MCS	*P* value
Case	36	41	
Gender (male/female)	21/15	21/20	0.532
Age (years)	40.22 ± 11.76	42.24 ± 11.01	0.439
Side (left/right)	19/17	22/19	1.000
Garden type			1.366
II	8	15	
III	16	20	
IV	12	6	
Time from injury to surgery (days)	2.83 ± 1.20	2.82 ± 1.20	0.988

**Table 2:** Comparison of postoperative follow-up between the PFLP and MCS groups.

	PFLP	MCS	*P* value
Intraoperative time	53.05 ± 12.77	47.78 ± 10.04	0.046
Intraoperative blood loss (ml)	36.66 ± 9.56	13.29 ± 7.12	<0.001
Fluoroscopy times	15.86 ± 3.53	23.26 ± 4.34	<0.001
Fracture healing (months)	4.82 ± 2.25	4.52 ± 1.76	0.533
All complications (nonunion/femoral neck necrosis/screw-out)	2	9	0.053
Femoral neck shorting			0.028
<5 mm	27	21	—
5–10 mm	6	11	—
>5 mm	3	9	—
Harris hip score	93.88 ± 7.26	87.92 ± 1.61	0.005

## Data Availability

The simulation experiment data used to support the findings of this study are available from the corresponding author upon request.
